# Antimicrobial Alkaloids from Marine-Derived Fungi as Drug Leads versus COVID-19 Infection: A Computational Approach to Explore their Anti-COVID-19 Activity and ADMET Properties

**DOI:** 10.1155/2022/5403757

**Published:** 2022-07-08

**Authors:** Sherouk Hussein Sweilam, Mohammed H. Alqarni, Fadia S. Youssef

**Affiliations:** ^1^Department of Pharmacognosy, College of Pharmacy, Prince Sattam Bin Abdulaziz University, Alkharj 11942, Saudi Arabia; ^2^Department of Pharmacognosy, Faculty of Pharmacy, Egyptian Russian University, Badr, Suez Road, 11829 Cairo, Egypt; ^3^Department of Pharmacognosy, Faculty of Pharmacy, Ain-Shams University, Abbasia, Cairo 11566, Egypt

## Abstract

Therapeutic strategies based upon enzyme inhibition have recently gained higher attention in treating hazardous ailments. Herein, the potential use of seventy-two antimicrobial alkaloids isolated from marine-derived fungi to fight COVID-19 infection *via* inhibition of SARS-CoV-2 lethal virus was performed using *in silico* analyses. Molecular modelling was performed to assess their enzyme inhibitory potential on the main protease SARS-CoV-2 M^Pro^, 3-chymotrypsin-like protease SARS-CoV-2 3CL^pro^, and papain-like protease SARS-CoV-2 PL^pro^ using Discovery Studio 4.5. Validation of the docking experiments was done by determination of RMSD (root mean square deviation) after redocking the superimposition of the cocrystalized ligands. Results showed that gymnastatin Z **(72)** showed the best fitting score in SARS-CoV-2 M^Pro^ and SARS-CoV-2 3CL^pr^ active sites with ∆G equal −34.15 and −34.28 Kcal/mol, respectively. Meanwhile, scalusamide C **(62)** displayed the highest fitting within SARS-CoV-2 PL^pro^ active sites (∆*G* = −26.91 Kcal/mol) followed by eutypellazine M **(57)**. ADMET/TOPKAT prediction displayed that eutypellazine M and scalusamide C showed better pharmacokinetic and pharmacodynamic properties. Gymnastatin Z is safer showing better toxicity criteria and higher rat oral LD_50_ and rat chronic LOAEL (lowest observed adverse effect level). Chemometric analysis using principle component analysis (PCA) based on the binding energies observed for the compounds with respect to the three tested enzymes revealed the clustering of the compounds into different clusters. Eutypellazine M, scalusamide C, and gymnastatin Z appear in one cluster due to their closeness in activity. Thus, these compounds could serve as promising SARS-CoV-2 enzymes inhibitors that could help in alleviation of COVID-19 infection. Further investigations are recommended to confirm the results of molecular modelling.

## 1. Introduction

The oceans constitute unique mines that offer a wide array of naturally occurring compounds derived mainly from marine organisms and their accompanied microorganisms [1]. As a result of evolution of infectious diseases and the subsequent appearance of resistance microbes *versus* the currently used anti-infectious agents, the marine resources may afford novel antimicrobial entities [2]. They could serve as promising leads combating viral, bacterial, fungal, and parasitic infections as well [3, 4]. Many naturally occurring marine products have successfully proceeded to the final stage of clinical trials; meanwhile others act as promising candidates for preclinical assessment [5]. Marine-derived fungal metabolites are characterized by favorable physicochemical behavior, oral bioavailability, and relative safety with respect to synthetic agents. This greatly highlights the considerable importance of these metabolites in the formulation of promising efficient pharmaceutical dosage forms that encourages us to carry out this study [6, 7].

The presence and dissemination of viral infections currently produce great distress as viral infections cause major health hazards. It is noteworthy to highlight that many antiviral leads *versus Herpes simplex* virus (HSV), influenza A (H1N1), and human immunodeficiency viruses (HIV) were isolated from marine sources [8]. Spongothymidine as well as spongouridine nucleosides isolated from *Tethya crypta* marine sponges led to Ara-A synthesis, an FDA approved antiviral drug that effectively prohibited viral DNA synthesis. Ara-A is converted into adenine arabinoside triphosphate that prohibits DNA polymerase and inhibits DNA synthesis of *Varicella zoster*, *Herpes*, and *Vaccinia* viruses. The clinical utilization of this compound has been used for the curing *Herpes* virus infection but was replaced by acyclovir (Zovirax) [9].

At the end of December 2019, patients possessing pneumonia of unidentified cause had spread in Wuhan, China. This was proved to be a novel coronavirus strain that triggered this fatal respiratory disease [10, 11]. This virus was termed severe acute respiratory syndrome-related coronavirus and abbreviated by SARS-CoV-2. On 12^th^ March 2020, coronavirus disease 2019 (COVID-19) has been ascertained in 125,048 patients all over the globe displaying about 3.7% mortality rate in comparison to influenza that showed less than 1% mortality rate [12]. Meanwhile, on 16 April, this lethal virus rapidly invaded 185 different countries and seriously infected more than 2,000,000 patients resulting in 130,000 deaths [10, 11, 13]. Besides, patients who suffer from severe COVID-19 also experienced cytokine storm syndrome. This is characterized by hyperinflammation, secondary hemophagocytic lymphohistiocytosis, continuous fever, cytopenias, hyperferritinemia, and pulmonary involvement that resulted in acute respiratory distress syndrome [10, 11]. Thus, searching for effective treatments to combat this pandemic is felt mandatory worldwide. This required the discovery of novel therapeutics comprising mainly vaccines and antivirals which target different viral proteins.

It is noteworthy to highlight that many researches have recently tried to use active constituents derived from natural products to combat COVID-19 infection guided by screening their activities using *in silico* studies [14–21].

As therapeutic strategies based upon enzyme inhibition have recently gained higher attention in treating hazardous ailments, thus in this study alkaloids from marine-derived fungal strains with antimicrobial potential reported in literature were collected based upon the authors' previous survey and published reviews [22, 23]. Around 72 alkaloid metabolites from *Arthrinium, Aspergillus, Eurotium, Curvularia*, *Eutypella, Dichotomomyces, Fusarium, Neosartorya*, *Penicillium, Paecilomyces, Stagonosporopsis*, *Thielavia, Pseudallescheria*, and *Westerdykella* specie*s* were found to display antimicrobial activities. The potential use of these diverse alkaloids to combat COVID-19 infection *via* inhibition of SARS-CoV-2 lethal virus was performed *via in silico* analyses. Molecular modelling was performed on three important enzymes which form crucial targets to prohibit SARS-CoV-2 replication, namely, main protease SARS-CoV-2 M^Pro^, 3-chymotrypsin-like protease SARS-CoV-2 3CL^pro^, and papain-like protease SARS-CoV-PL^pro^. Furthermore, ADMET/TOPKAT (absorption, distribution, metabolism, excretion, and toxicity) prediction was done on the compounds that showed the highest activity towards the examined enzymes to explore their pharmacokinetic, pharmacodynamic, and toxicity properties. This was done in an effort to explore lead compounds that could serve as promising entities to help in solving the present health crises. In addition, chemometric analysis was performed based on the fitting score values aiming to correlate compounds with similar activity.

## 2. Materials and Methods

### 2.1. Selection of Compounds Used in This Study

A comprehensive literature survey was performed by the authors focusing on the biological activities and chemical properties of alkaloids isolated from marine associated twenty-seven fungal genera. These fungal genera comprise *Acrostalagmus, Aspergillus, Arthrinium, Curvularia, Chaetomium, Coniothyrium, Cladosporium*, *Eurotium*, *Dichotomomyces, Eutypella*, *Fusarium, Exophiala*, *Hypocrea*, *Microsphaeropsis*, *Neosartorya, Microsporum*, *Nigrospora, Paecilomyces, Pleosporales, Penicillium*, *Scedosporium, Pseudallescheria, Stagonosporopsis, Scopulariopsis*, *Westerdykella, Xylariaceae*, and *Thielavia* [22, 23]. Around 514 alkaloid metabolites were isolated and identified *via* various chromatographic and spectroscopic techniques. They were additionally ascertained using High Resolution Mass Spectrometry together with Mosher reactions for further confirmation of the stereochemistry. Around 72 alkaloid metabolites were reported to possess antiviral, antibacterial, and antifungal activities which were selected to be the target of our study. Data were collected from PubMed (https://www.ncbi.nlm.nih.gov/pubmed/), sciFinder (https://scifinder.cas.org/scifinder/login), and Web of Knowledge (https://www.webofknowledge.com).

### 2.2. *In silico* Studies

Molecular modelling was performed on SARS-CoV-2 M^Pro^ (PDB ID: 6LZE; 1.50 A°), SARS-CoV-2 3CL^pro^ (PDB ID: 6M2N; 2.20 A°), SARS-CoV-PL^pro^ (PDB ID: 4OW0; 2.10 A°), and ACE2 (PDB ID: 1R4L; 3.00 A°) using Discovery Studio 4.5 (Accelrys Inc., San Diego, CA, USA) applying C-Docker protocol as previously discussed [24–26]. The X-ray crystal structures of the examined proteins were obtained from protein data bank (https://www.pdb.org) in PDB format. This was done for seventy-two compounds of the identified alkaloids that previously showed to exhibit significant antimicrobial and antiviral activities.

#### 2.2.1. Validation of Molecular Docking Studies Using Redocking and Superimposition

Molecular docking validation was done for all the performed docking experiments through performing a comparison between the alignments of the most stable docking poses of the lead compound together with the lead conformer cocrystalized with the respective enzyme from PDB. The value of RMSD (root mean square deviation) is utilized to ascertain the docking experiment validity and gives an indication to the ability of prediction of the binding affinity of new ligands.

#### 2.2.2. Performing Molecular Docking Studies

The structure for each enzyme was prepared *via* adopting the default protocol of Discovery Studio 4.5 (Accelrys Inc., San Diego, CA, USA) [24, 27, 28]. This occurs in several steps starting with removal of water molecules, adding of hydrogen atoms accompanied by cleansing the structure of the protein from undesired interactions. CHARMm was employed as the forcefield; however MMFF94 was adopted for partial charge calculation that subsequently was followed by minimizing the added hydrogen in 2000 steps. Determination of the binding center was accomplished depending upon the data reported approaching the catalytic domain of the targeted protein. ChemDraw 13.0 was used to construct the 2D structures of the compounds that consequently were saved as PDB files. The default protocol for ligand preparation was used to prepare the 3D structures of the compounds for docking experiments. Docking was then performed for the prepared structure within the active centers of the energy-minimized protein employing default parameters in C-Docker protocol. CHARMm force ﬁeld was chosen and the binding energy (ΔG) was computed using distance dependent dielectric implicit solvation model for the chosen docking poses. Calculation of (Δ*G*) in Kcal/mol was performed using the following equation:

(1) $$\begin{array}{c} \Delta G_{\text{binding}}=E_{\text{complex}}-\left(E_{\text{protein}}+E_{\text{ligand}}\right), \end{array}$$

where Δ*G*_binding_ is the ligand-protein interaction binding energy, *E*_complex_ is the potential energy for the complex of protein bound with the ligand, *E*_protein_ is the protein potential energy alone, and *E*_ligand_ is the ligand potential energy alone.

#### 2.2.3. ADMET/TOPKAT Prediction

ADMET/TOPKAT (absorption, distribution, metabolism, excretion, and toxicity) prediction was done on the compounds that showed the highest activity towards the examined enzymes together with the cocrystalized ligands using Discovery Studio 4.5 (Accelrys Inc., San Diego, CA, USA). Human intestinal absorption, blood brain barrier penetration (BBB), aqueous solubility, hepatotoxicity level, plasma protein binding prediction (PPB), and cytochrome P450 (2D6) were selected as ADMET descriptors. However, Ames mutagenicity, carcinogenic effect female and male rat FDA, rat oral LD_50_, and rat chronic LOAEL in addition to eye and dermal irritancy were selected as toxicity parameters [29].

### 2.3. Chemometric Analysis

Chemometric analysis using principle component analysis (PCA) as unsupervised pattern recognition technique was done based on the binding energies observed for the compounds with respect to the three tested proteins using CAMO's Unscrambler® X 10.4 software (Computer-Aided Modeling, As, Norway) [26].

## 3. Results and Discussion

### 3.1. Diverse Alkaloids Identified from Marine-Derived Fungal Strains Showing Antimicrobial Activities

Around 72 alkaloids isolated from marine associated fungal strains belonging to *Arthrinium, Aspergillus, Eurotium, Curvularia, Eutypella, Dichotomomyces,, Fusarium, Neosartorya, Penicillium, Paecilomyces, Stagonosporopsis, Thielavia, Pseudallescheria*, and *Westerdykella* were reported to possess antimicrobial activities [22, 23]. These include arthpyrones F-I **(1–4)** and apiosporamide **(5)** isolated from *Arthrinium* [30]. Additionally, *Aspergillus* species act as a rich source of alkaloids with anti-infective properties such as fumitremorgin C **(6),** fumiquinazoline C **(7)**, 12,13-dihydroxy fumitremorgin C (**8)**, fumiquinazoline G **(9)**, fumigatoside E **(10)**, fumigatoside F **(11)**, epi-aszonalenin A **(12)**, versicoloids A and B **(13-14)**, aspergicin **(15)**, stephacidin A **(16)**, 7*α*,14-dihydroxy-6*β*-p-nitrobenzoylconfertifolin **(17)**, 9*α*,14-dihydroxy-6*β*-p-nitrobenzoylcinnamolide **(18),** 3-((1-hydroxy-3-(2-methylbut-3-en-2-yl)-2-oxoindolin-3yl)methyl)-1-methyl-3,4-dihydrobenzo[e] [1, 4] diazepine-2,5-dione **(19),** cytochalasin Z17 **(20),** and gliotoxin **(21)** [30–37]. Moreover, curvulamine **(22)** obtained from *Curvularia* species as well as scequinadoline A **(23)** isolated from *Dichotomomyces* revealed potent antimicrobial activity [38].

Meanwhile, *Eurotium* isolated from marine sources contains alkaloids that showed antimicrobial activity including neoechinulin B **(24)**, cristatumin A **(25)**, rubrumazines A-C **(26–28)**, compounds **(29–40)**, isoechinulin A **(41)**, rubrumline D (42), variecolorine O (43), and neoechinulin C **(44)** [39, 40]. New compounds, eutypellazines A-M **(45–57)**, obtained from *Eutypella*, are potent antimicrobial fungal metabolites [41]. Oxysporizoline **(58)**, a new polycyclic quinazoline alkaloid isolated from *Fusarium*, [42] and varioxepine A **(59)** isolated from the marine associated fungi *Paecilomyces*, exhibited a potent antimicrobial activity [43]. *Penicillium* is a popular source of marine associated fungi rich in bioactive alkaloids particularly showing antimicrobial properties. These are scalusamides A-C **(60–62)**, penipanoid A **(63)** and C **(64)**, raistrickindole A **(65)**, raistrickin **(66)**, brevianamide F **(67)**, *α*-cyclopiazonic acid **(68),** and terretrione A **(69)** [44, 45]. Didymellamide A **(70)** from *Stagonosporopsis* [46] and thielaviazoline **(71)** from *Thielavia*, a marine associated fungus, are potent antimicrobial agents [47]. Gymnastatin Z (**72**), a new tyrosine-derived alkaloid, was isolated from *Westerdykella dispersa* and displayed moderate antimicrobial effect [48]. The structures of all the antimicrobial alkaloids isolated from the previously mentioned fungi are depicted in Figures 1–3.

### 3.2. *In silico* Studies

SARS-CoV-2 reveals a genome greatly similar to *beta*-coronaviruses comprising a replicase region containing a replicase complex (orf1ab) that produces nonstructural proteins (nsps), a 5' -untranslated region (UTR), a structural region composed of an envelope protein (E) gene, a spike protein (S) gene, a nucleocapsid protein (N) gene, and a membrane protein (M) gene in addition to 3'—UTR and multiple unidentified non-structural open reading frames [11]. Although SARS-CoV-2 was classified as *beta*-coronaviruses, it shows certain similarities and other differences from MERS-CoV and SARS-CoV genome. Besides, during genome transcription, *beta*-coronaviruses generate a polypeptide (about 800 kDa) that undergoes proteolytic cleavage performed by main protease (M^Pro^), papain-like protease (PL^pro^), and 3-chymotrypsin-like protease (3CL^pro^) to produce different proteins at 11 specific sites which are crucial for viral replication. Thus, targeting these enzymes may act as important therapeutic strategies to inhibit SARS-CoV-2 [11]. Thus, herein shedding the light on the potential use of diverse antimicrobial alkaloids derived from marine fungi as SARS-CoV-2 M^Pro^, papain-like protease (PL^pro^), and SARS-CoV-2 3CL^pro^ inhibitors was adopted. This was performed *via* molecular modelling study as future perspectives in an effort to inhibit this virus and combat COVID-19 infection. Molecular modelling was performed on SARS-CoV-2 M^Pro^ (PDB ID: 6LZE; 1.50 Å), SARS-CoV-2 3CL^pro^ (PDB ID: 6M2N; 2.20 Å), and SARS-CoV-2 PL^pro^ (PDB ID: 7LOS; 2.9 Å) using Discovery Studio 4.5 (Accelrys Inc., San Diego, CA, USA) employing C-Docker protocol as previously discussed [24–26]. This was done for seventy-two compounds of previously identified alkaloids that previously showed significant antimicrobial and antiviral activities. The structures of the three targeted proteins were illustrated in Figure 4.

#### 3.2.1. Validation of the Molecular Docking Experiments

Validation experiments showed a perfect alignment between the docking pose of the lead compounds that showed the highest fitting and the lead conformers that are cocrystalized with their respective enzymes. They displayed RMSD values of 1.30, 1.75, and 2.02 Å for SARS-CoV-2 PL^pro^, SARS-CoV-2 M^Pro^, and SARS-CoV-2 3CL^pro^, respectively. Thus, it perfectly ascertained the validity of the docking experiment as shown in Figure 5 [49].

#### 3.2.2. Molecular Modelling Studies

Molecular modelling of the seventy two selected compounds revealed that gymnastatin Z **(72)** showed the best fitting score in SARS-CoV-2 M^Pro^ and SARS-CoV-2 3CL^pr^ active sites followed by scalusamide C **(62)** and eutypellazine M **(57);** meanwhile scalusamide C **(62)** displayed the highest fitting within SARS-CoV-2 PL^pro^ active sites followed by gymnastatin Z **(72)** and eutypellazine M **(57).** They showed binding energies (∆ *G*) equal to −34.15, −29.34, and -25.44 Kcal/mol, respectively, for SARS-CoV-2 M^Pro^, −24.29, −26.91, and −22.21 Kcal/mol, respectively, for SARS-CoV-2 PL^pro^, whereas they showed ∆*G* of −34.28, −32.73, and −31.5237 Kcal/mol, respectively, for SARS-CoV-2 3CL^pr^. Thus, in this aspect, they showed superior activity in comparison to the main SARS-CoV-2 M^Pro^ ligand (FHR/PRD_002347 (∼{N}-[(2∼{S})-3-cyclohexyl-1-oxidanylidene-1-[[(2∼{S})-1-oxidanylidene-3-[(3∼{S})-2-oxidanylidenepyrrolidin-3-yl] propan-2-yl]amino]propan-2-yl]-1∼{H}-indole-2-carboxamide) (∆*G* = −4.60 Kcal/mol) and that of SARS-CoV-2 PL^pro^ ligand: Y975-(azetidin-3-ylamino)-2-methyl-∼{N}-[(1∼{R})-1-[3-[5-[[[(3∼{R})-oxolan-3-yl]amino]methyl]thiophen-2-yl]phenyl]ethyl]benzamide (∆*G* = −4.08 Kcal/mol) downloaded with the protein from PDB. Meanwhile, they approach that of the main SARS-CoV-2 3CL^pr^ ligand: 3WL (5,6,7-trihydroxy-2-phenyl-4H-chromen-4-one) (∆*G* = −34.67 Kcal/mol) downloaded with the protein from PDB as revealed in Table 1.

The significant fitting of gymnastatin Z **(72)** at the binding site of SARS-CoV-2 M^Pro^ can be interpreted by means of producing multiple bonds with the amino acid moieties existing in the active center. This was evidenced by three H-bonds formed with His 163, Glu 166, and Phe 140 together with the formation of one *π*-alkyl interaction with Cys 145, alkyl-alkyl interactions with Pro 168 and Met 49, and Van der Waals interaction with many amino acid groups present in the active pocket (Figure 6(a)). Regarding scalusamide C **(62),** similarly it forms multiple bonds comprising two H-bonds with Gln 192 and Met 165, alkyl-alkyl interactions with Met 49 and His 163 in addition to C-H bond with Glu 166, and many Van der Waals interactions (Figure 7(a)). However, eutypellazine M **(57)** forms conventional H-bond between the OH group in the compound and the amino acid Gln 189, *π*-sulfur bond between the aromatic benzene ring and Cys 145, and *π*-alkyl bond between Met 165 and the benzene ring together with the presence of Van der Waals interaction with most of the aminoacid groups existing in the active site (Figure 8(a)). Meanwhile, the main SARS-CoV-2 M^Pro^ ligand showed conventional H-bond with Glu 166, alkyl bond with Cys 145, *π*-alkyl bond with Pro 168, and C-H bond with His 164, Gln 189, His 41, and Asn 142 in addition to Van der Waals interaction with the amino acid residues present in the active site (Figure 9(a)).

Concerning SARS-CoV-2 PL^pro^, gymnastatin Z **(72)** forms one H-bond with Gly 266 in addition to two *π*-alkyl interactions with Tyr 268 and Pro 248 together with one alkyl interaction with Pro 248 and Van der Waals interaction (Figure 6(b)). However, scalusamide C **(62)** showed the highest fitting score evidenced by the presence of one alkyl interaction with Pro 248, four C-H interactions with Asp 164, Pro 247, and Pro248, and Van der Waals interaction (Figure 7(b)). Additionally, eutypellazine M **(57)** forms one conventional H-bond with Arg 166, *π*-*π* stacked bond with Tyr 268, and C-H bond with Pro 248, Asp164, and Arg 166 with many Van der Waals bonds (Figure 8(b)). Meanwhile, the main SARS-CoV-2 PL^pro^ ligand forms four H-bonds with Glu 167, Asp 164, Gln 269, and Gly 266, one *π*-*π* bond with Tyr 268, two *π*-alkyl interactions with Pro 248 and Tyr 264, 2 alkyl interactions with Pro 248 and Leu 162, and four C-H bonds with Glu 167, Gly 266, and Pro 248 and *π*-sulfur bond with Tyr 264 (Figure 9(b)).

Regarding SARS-CoV-2 3CL^pr^, gymnastatin Z **(72)** also exerted the highest fitting that relied upon the presence of three H-bonds with His 41, His 164, and Glu 166 and alkyl-alkyl interactions with Met 49, Cys 44, Pro 52, and His 41, whereas the *π*-*δ* bond is formed between Asn 142 and the aromatic moiety of the phenyl ring (Figure 6(c)). Scalusamide C **(62)** is also tightly bound to the active site due to the presence of one H-bond with Glu 166, one C-H bond with Met 165, and alkyl interactions with Cys 145, His 41, Met 49, Leu 167, and Pro 168 (Figure 7(c)). Eutypellazine M **(57)** also revealed the best fitting score that is manifested by its firm binding at the active site via the formation of several bonds with the amino acid residues present at the active sites. They are 2 conventional H-bonds with His 164 and His 41, *π*-sulfur bond with Cys 44, *π*-*π* T-shaped bond with His 41, and Van der Waals interaction with most of the amino acid groups at the active center, *π*-alkyl bond with Met 49 and Cys145 (Figure 8(c)). However, main SARS-CoV-2 3CL^pr^ ligand: 3WL formed 4 H-bonds with Leu 141, Ser 144, Gly 143, and Cys 145, *π*-sulfur bond with Cys 145, *π*-alkyl bond with Met 49, *π*-*π* stacked bond with His 41, and C-H bond with His 163 together with Van der Waals interaction with most of the amino acid groups at the active center (Figure 9(c)). The presence of gymnastatin Z in the active pocket of SARS-CoV-2 M^Pro^ (A), SARS-CoV-2 PL^pro^ (B), and SARS-CoV-2 3CL^pr^ (C) active sites showing regions of hydrogen bond formation, hydrophobicity regions, and ionizable regions is illustrated in Figure 10. Additionally, the compounds that showed the highest fitting within the previously mentioned enzymes, namely, gymnastatin Z **(72),** scalusamide C **(62),** and eutypellazine M **(57),** were docked within the active sites of angiotensin-converting enzyme 2 ACE2 where they also showed a pronounced fitting with ∆*G* of −40.90, −37.74, and −52.28 kcal/mol, respectively. Eutypellazine M **(57)** that showed the best fitting with the active site forms different bonds evidenced by the formation of four H-bonds with Arg273, Glu402, His378, and Tyr515, one *π*-alkyl bond with Pro346 in addition to one C-H bond with Ala348, and many Van der Waals interactions.

#### 3.2.3. ADMET/TOPKAT Prediction

ADMET/TOPKAT prediction was evaluated for eutypellazine M **(57)**, scalusamide C **(62),** and gymnastatin Z **(72),** as well as the cocrystalized ligands with the examined proteins in order to determine their pharmacokinetic and pharmacodynamic characters (Table 2). Both eutypellazine M and scalusamide C revealed good human intestinal absorption level, good solubility level, and certain BBB level and thus they lie within the 99% absorption ellipse as well as the 99% BBB confidence ellipse as shown in ADMET plot (Figure 11). Meanwhile, gymnastatin Z showed low human intestinal absorption level with possible solubility and undefined BBB level and thus in ADMET plot it is found outside the 99% BBB confidence ellipse. Regarding plasma protein binding level that is crucial in the determination of pharmaceutical activity as it controls the concentration of free drug, gymnastatin Z displayed less than 90% PPB whereas both eutypellazine M and scalusamide C showed more than 90% binding. Regarding the toxicity parameters, eutypellazine M, scalusamide C, and gymnastatin Z are nonhepatotoxic, nonmutagen, and noncarcinogen to both male and female rat FDA. They also caused no cytochrome P450 2D6 (CYP2D6) inhibition that is involved in the metabolism of many xenobiotics so its inhibition may be the cause of uncontrolled drug-drug interactions. Rat oral LD_50_ was 0.28, 1.35, and 1.16 g/kg.bw for eutypellazine M, scalusamide C, and gymnastatin Z, respectively; meanwhile 0.03, 0.08 and 0.18 g/kg.bw were the values for rat chronic LOAEL (lowest-observed-adverse-effect level) for them, respectively. Regarding ocular and dermal irritation, gymnastatin Z showed mild skin irritation with no eye irritation in contrast to eutypellazine M that showed severe eye irritation and no dermal irritancy. From ADMET/TOPKAT prediction, it can be concluded that eutypellazine M **(57)** and scalusamide C **(62)** showed better pharmacokinetic and pharmacodynamic properties when compared to gymnastatin Z; however gymnastatin Z is safer showing better toxicity criteria and higher rat oral LD_50_ as well as rat chronic LOAEL in addition to better inhibitory activity to the tested enzymes as revealed from the docking scores. Thus, it should be subjected to certain semisynthetic treatment to improve its pharmacokinetic and pharmacodynamic properties to be suitable for incorporation in pharmaceutical dosage forms without affecting its activity or safety.

### 3.3. Chemometric Analysis

Chemometric analysis using principle component analysis (PCA) as unsupervised pattern recognition technique was done based on the binding energies observed for the compounds with respect to the three tested proteins. Compounds are clustered into four main clusters taking different colors and symbols as revealed in Figure 12 with compounds similar in activity for the three tested proteins gathered in one cluster. Moreover, eutypellazine M **(57)**, scalusamide C **(62),** and gymnastatin Z **(72**) are gathered together in a subcluster lying in the left lower quadrant near to main axis of PC2 due to their closeness in activity. In contrast, *epi*-aszonalenin A **(12)** and cytochalasin Z17 **(20)** are outliers that mainly relied upon their completely different values particularly towards SARS-CoV-PL^pro.^ This in turn reflects their ineffectiveness towards the examined enzymes. Chemometric analysis acts as a simple tool that makes it easier to recognize the variation and closeness in activities among the tested chemical entities. The clustering of the different compounds based upon their ∆*G* towards the three tested proteins is illustrated in Figure 12.

## 4. Discussion

Molecular modelling has been adopted by many researchers to screen the possibility of using the active constituents derived from natural products to combat COVID-19 infection. Many viral enzymes serve as promising targets for the discovery of new drug leads combating COVID-19 infection. This includes main protease (M^Pro^), papain-like protease (PL^pro^), 3-chymotrypsin-like protease (3CL^pro^), angiotensin-converting enzyme 2 (ACE2), and RNA-dependent RNA polymerase (RdRp) [14–16]. The structural protein, the viral S protein, and angiotensin-converting enzyme 2 receptor (host receptor) may particularly act as an important therapeutic target in the virus eradication. S protein allows viral infection through angiotensin-converting enzyme 2 (ACE-2) receptor recognition and membrane fusion [50]. Components that affect SARS CoV-2 serve as a perfect strategy for the discovery of lead drug entities combating COVID-19 infection.

Like MERS and SARS, the genome of SARS CoV-2 possesses two open reading frames which are ORF1a and ORF1ab that perfectly help in the translation of two viral polyproteins pp1a and pp1ab. They are overlapped together and crucial in the replication and transcription of the virus. Consequently, functional polypeptides are obtained from two viral polyproteins via proteolytic processing performed by papain-like proteinase (PL^pro^) [51]. SARS-CoV PLpro and SARS-CoV-2 PLpro showed 82.9% sequence identity; meanwhile it revealed 100% sequence identity for the binding site reported to accommodate small molecules in SARS-CoV. Additionally, they revealed comparable fold with no deviation in backbone conformations and thus it could be also used while screening compounds as possible SARS-COV-2 inhibitors [52]. Moreover, PLpro and 3CLpro are mainly responsible for the cleavage of three and eleven sites, respectively, within the viral genome, and thus the latter is termed by main protease or M^pro^ because it cleaves more sites. Furthermore, M^pro^ plays a critical function in polyprotein processing and virus maturation, and thus it is regarded as a considerable target for designing antiviral drugs against SARS CoV-2. Adopting computational studies, researchers have discovered plenty of small molecules comprising HIV and malaria drugs as potent SARS CoV-2 protease inhibitor. Additionally, many antiviral bioactive constituents derived from Moroccan and Indian medicinal plants such as digitoxigenin, arjunglucoside-I, crocin, carnosol, *β*-eudesmol, and rosmanol are prospected to be promising SARS CoV-2 M^pro^ inhibitors [51].

Regarding marine-derived compounds, *in silico* studies revealed the effectiveness of many drug entities *versus* SARS CoV-2 various enzymes. Callophysin A isolated from red alga *Callophycus oppositifolius* displayed a potent SARS-CoV-2 3CL^pr^ inhibitory potential. This was achieved via the formation of hydrogen bonds, salt bridge, and hydrophobic interactions with the amino acid moieties at the catalytic sites (Cys145 and His41) [53]. Additionally, *in silico* study performed on marine compounds possessing antiviral potential revealed that pyrrole carboxamide, acyl indole, and compounds having a flavonoid nucleus displayed the highest docking scores while binding to spike glycoprotein, RNA polymerase, and main protease of SARS-CoV-2 active sites. Besides, debromosceptrin and sceptrin revealed complete alignment with the ligand cocrystalized with main protease. Meanwhile, thalassoilin (A-B) displayed the best fitting with all the tested proteins [54].

Besides, a study carried out by Ibrahim et al. revealed that bis([1, 3]dioxolo)pyran-5-carboxamide derivatives showed significant activity against SARS-CoV-2 M^pro^ and are ready to be examined for *in vitro* inhibition against SARS-CoV-2 [55]. Meanwhile, canthin-6-one 9-O-*beta*-glucopyranoside showed the highest binding affinity and less binding energy with both PL^pro^ and M^pro^/3CL^pro^ proteases and thus it can be used as a potential natural drug against COVID-19 protease [56]. Furthermore, phytochemicals of the plant *Boerhavia diffusa* such as *β*-ecdysone, bioquercetin, biorobin, boeravinone J, boerhavisterol, kaempferol, liriodendrin, quercetin, and *trans*-caftaric acid were docked to SAR-CoV-2 main protease. Biorobin, bioquercetin, and boerhavisterol showed the best binding energies and were found to be favorable for an efficient docking and resultant inhibition of the viral main protease [57].

Herein, molecular modelling of 72 antimicrobial alkaloids derived from fungi performed on the main protease SARS-CoV-2 M^Pro^, 3-chymotrypsin-like protease SARS-CoV-2 3CL^pro^, and papain-like protease SARS-CoV-PL^pro^ showed that gymnastatin Z exhibited the best fitting on SARS-CoV-2 M^Pro^, SARS-CoV-2 3CL^pr^, and SARS-CoV-PL^pro^ followed by scalusamide C and eutypellazine M. The significant fitting of these compounds can be interpreted by the means of formation of several bonds with the amino acid moieties existing in the active pocket as revealed by 2D and 3D binding modes. The evident variation among the compounds with respect to the presence or absence of functional moieties as well as the size of the molecule even the length of the substituted alkyl chains effectively contributes to the activity of the tested metabolites. Increasing the complexity of the structure as in eutypellazine series reduces the activity that is evidenced by the high activity of eutypellazine M compared to eutypellazine A. ADMET/TOPKAT prediction displayed that eutypellazine M and scalusamide C possess better pharmacokinetic and pharmacodynamic properties. However, gymnastatin Z is safer showing better toxicity criteria and higher Rat oral LD_50_ as well as rat chronic LOAEL in addition to better inhibitory activity on the tested enzymes as revealed from the docking scores. Thus, gymnastatin Z should be subjected to certain treatment to improve its pharmacokinetic and pharmacodynamic properties to be suitable for incorporation in pharmaceutical dosage forms without affecting its activity or safety. Thus, these compounds could serve as promising lead entities with high enzyme inhibitory potential that could inhibit SARS-CoV-2. Further investigations are required to confirm the results of molecular modelling. Thus, computational studies performed on natural occurring compounds could help in searching for new lead entities to solve the crisis of COVID-19 with low cost in comparison to *in vitro* and *in vivo* assays. However, that revealed activity should be subjected to further in depth *in vitro* and *in vivo* studies followed by preclinical trials to confirm the obtained results.

## 5. Conclusions

Marine-derived fungal strains constitute a promising source of bioactive alkaloids. Seventy-two alkaloid metabolites showed antimicrobial activities as recently collected from literature. Molecular modelling of these compounds performed after validation of the docking experiments revealed that gymnastatin Z showed the best fitting score on SARS-CoV-2 M^Pro^, SARS-CoV-PL^pro^, and SARS-CoV-2 3CL^pr^. This is followed by scalusamide C and eutypellazine M. ADMET/TOPKAT prediction displayed that eutypellazine M and scalusamide C showed better pharmacokinetic and pharmacodynamic properties. However, gymnastatin Z is safer showing better toxicity criteria; thus, it could be subjected to certain treatment to improve its pharmacokinetic and pharmacodynamic properties to be suitable for incorporation in pharmaceutical dosage forms without affecting its activity or safety. Additionally, they were clustered close to each other as manifested by the PCA analysis. Thus, these compounds could serve as promising enzyme inhibitors for drug discovery of successful pharmaceutical products that could inhibit SARS-CoV-2 and overcome COVID-19 pandemic. However, further investigations *via in vitro* and *in vivo* studies are required to be conducted to confirm the results of molecular modelling.

## Figures and Tables

**Figure 1:** Diverse alkaloids identified from marine-derived fungal strains showing antimicrobial activities.

**Figure 2:** Diverse alkaloids identified from marine-derived fungal strains showing antimicrobial activities (cont'd).

**Figure 3:** Diverse alkaloids identified from marine-derived fungal strains showing antimicrobial activities (cont'd).

**Figure 4:** The ribbon structure of the three targeted proteins, SARS-CoV-2 M^Pro^ (a), SARS-CoV-2PL^pro^, (b) and SARS-CoV-2 3CL^pro^ (c) downloaded from the protein data bank.

**Figure 5:** Validation of the docking experiments for SARS-CoV-2 M^Pro^ (a), SARS-CoV-2 PL^pro^ (b), and SARS-CoV-2 3CL^pro^ (c).

**Figure 6:** 2D and 3D binding modes of the gymnastatin Z **(72)** in SARS-CoV-2 M^Pro^ (a), SARS-CoV-2PL^pro^ (b), and SARS-CoV-2 3CL^pr^ (c) active sites.

**Figure 7:** 2D and 3D binding modes of the scalusamide C **(62)** in SARS-CoV-2 M^Pro^ (a), SARS-CoV-PL^pro^ (b), and SARS-CoV-2 3CL^pr^ (c) active sites.

**Figure 8:** 2D and 3D binding modes of the eutypellazine M **(57)** in SARS-CoV-2 M^Pro^ (a), SARS-CoV-2 PL^pro^ (b), and SARS-CoV-2 3CL^pr^ (c) active sites.

**Figure 9:** 2D and 3D binding modes of the respective ligands in SARS-CoV-2 M^Pro^ (a), SARS-CoV-2 PL^pro^ (b), and SARS-CoV-2 3CL^pr^ (c) active sites.

**Figure 10:** The presence of gymnastatin Z in the active pocket of SARS-CoV-2 M^Pro^ (a), SARS-CoV-2 PL^pro^ (b), and SARS-CoV-2 3CL^pr^ (c) active sites showing regions of hydrogen bond formation, hydrophobicity regions, and ionizable regions.

**Figure 11:** ADMET Plot for bioactive compounds, eutypellazine M **(57)**, scalusamide C **(62),** and gymnastatin Z **(72)** and the cocrystalized ligands with the examined proteins showing the 95% and 99% confidence limit ellipses corresponding to the blood brain barrier (BBB) and the human intestinal absorption models; eutypellazine M **(57)**, (triangle); scalusamide C **(62)** (filled square); and gymnastatin Z **(72)**, (star) in ADMET_AlogP98.

**Figure 12:** PCA score plot performed based on the binding energies observed for the compounds with respect to the three tested proteins. Compounds are numbered as given in Table 1. The black arrow indicates the presence of eutypellazine M **(57)**, scalusamide C **(62),** and gymnastatin Z **(72)** close to each other in a subcluster.

**Table 1:** Binding energies (∆*G*) of the docked compounds expressed in kcal/mole using *in silico* studies within the active centers of SARS-CoV-2 M^Pro^, SARS-CoV-2PL^pro^, and SARS-CoV-2 3CL^pr^.

Compound	Genus	SARS-CoV-2 M^Pro^	SARS-CoV-2 PL^pro^	SARS-CoV-2 3CL^pr^
Arthpyrone F **(1)**	*Aspergillus*	20.01	26.33	12.49
Arthpyrone G **(2)**	*Aspergillus*	47.11	47.43	44.89
Arthpyrone H **(3)**	*Aspergillus*	21.01	29.33	14.49
Arthpyrone I **(4)**	*Aspergillus*	23.28	39.35	23.92
Apiosporamide **(5)**	*Aspergillus*	7.29	23.30	6.18
Fumitremorgin C **(6)**	*Aspergillus, Pseudallescheria*	5.12	12.48	4.36
Fumiquinazoline C **(7)**	*Aspergillus*	11.92	43.37	12.07
12,13-Dihydroxy fumitremorgin C (**8)**	*Aspergillus, Pseudallescheria*	−5.12	−12.48	−4.36
Fumiquinazoline G **(9)**	*Aspergillus*	19.91	29.28	17.30
Fumigatoside E **(10)**	*Aspergillus*	2.57	4.77	6.28
Fumigatoside F **(11)**	*Aspergillus*	−1.57	2.77	−5.28
*epi*-Aszonalenin A **(12)**	*Aspergillus*	27.74	233.99	27.2962
Versicoloid A **(13)**	*Aspergillus*	−14.40	−6.18	−15.17
Versicoloid B **(14)**	*Aspergillus*	−10.39	−4.22	−12.12
Aspergicin **(15)**	*Aspergillus*	−12.43	−5.21	−14.19
Stephacidin A **(16)**	*Aspergillus*	23.86	29.94	23.69
Compound **(17)**	*Aspergillus*	18.25	20.25	20.25
Compound **(18)**	*Aspergillus*	24.49	22.05	20.66
Compound **(19)**	*Aspergillus*	0.12	21.08	0.95
Cytochalasin Z17**(20)**	*Aspergillus*	39.52	128.81	41.66
Gliotoxin **(21)**	*Aspergillus*	24.35	32.94	26.95
Curvulamine **(22)**	*Curvularia*	15.23	17.72	9.62
Scequinadoline A **(23)**	*Dichotomomyces*	−5.32	31.30	−10.14
Neoechinulin B **(24)**	*Eurotium*	−12.62	−12.99	−17.19
Cristatumin A **(25)**	*Eurotium*	−17.28	−14.32	−21.48
Rubrumazine A **(26)**	*Eurotium*	−20.945	10.63	−23.22
Rubrumazine B**(27)**	*Eurotium*	−21.11	10.37	−23.02
Rubrumazine C **(28)**	*Eurotium*	−20.334	−12.64	−22.96
Compound **(29)**	*Eurotium*	−13.83	−17.65	−18.81
Compound **(30)**	*Eurotium*	−2.41	6.93	−3.06
Compound **(31)**	*Eurotium*	−6.73	17.15	−3.05
Compound **(32)**	*Eurotium*	15.00	54.20	6.22
Compound **(33)**	*Eurotium*	−26.77	−9.58	−27.69
Compound **(34)**	*Eurotium*	−19.50	−10.22	−24.53
Compound **(35)**	*Eurotium*	18.16	67.10	22.15
Compound **(36)**	*Eurotium*	33.22	FD	30.89
Compound **(37)**	*Eurotium*	−19.24	−25.36	−21.94
Compound **(38)**	*Eurotium*	−15.36	−12.32	−21.52
Compound **(39)**	*Eurotium*	−6.69	26.60	−8.54
Compound **(40)**	*Eurotium*	−13.83	15.93	−1.76
Isoechinulin A **(41)**	*Eurotium*	−1.17	−0.52	−6.21
Rubrumline D **(42)**	*Eurotium*	−22.96	−3.98	−21.88
Variecolorine O **(43)**	*Eurotium*	−20.22	−21.52	−24.26
Neoechinulin C **(44)**	*Eurotium*	−2.17	3.17	15.50
Eutypellazine A **(45)**	*Eutypella*	34.07	59.98	36.55
Eutypellazine B **(46)**	*Eutypella*	41.54	52.74	42.17
Eutypellazine C **(47)**	*Eutypella*	30.37	59.19	31.74
Eutypellazine D **(48)**	*Eutypella*	17.54	63.22	15.50
Eutypellazine E **(49)**	*Eutypella*	27.24	12.27	23.06
Eutypellazine F **(50)**	*Eutypella*	17.83	12.58	17.47
Eutypellazine G **(51)**	*Eutypella*	21.80	9.57	24.47
Eutypellazine H **(52)**	*Eutypella*	30.28	7.70	30.27
Eutypellazine I **(53)**	*Eutypella*	−19.44	6.62	−23.38
Eutypellazine J **(54)**	*Eutypella*	−22.19	−6.84	−25.75
Eutypellazine K **(55)**	*Eutypella*	−24.46	−3.43	−28.53
Eutypellazine L **(56)**	*Eutypella*	−24.24	−6.01	−26.82
Eutypellazine M **(57)**	*Eutypella*	**−25.44**	**−22.21**	**−31.52**
Oxysporizoline **(58)**	*Fusarium*	FD	FD	FD
Varioxepine A **(59)**	*Paecilomyces*	FD	FD	FD
Scalusamide A **(60)**	*Penicillium*	−14.08	−19.86	−17.83
Scalusamide B **(61)**	*Penicillium*	−13.55	−21.52	−14.25
Scalusamide C **(62)**	*Penicillium*	**−29.34**	**−26.91**	**−32.73**
Penipanoid A **(63)**	*Penicillium*	11.34	9.65	6.96
Penipanoid C **(64)**	*Penicillium*	−13.92	−15.16	−18.17
Raistrickindole A **(65)**	*Penicillium*	−5.87	27.75	−9.07
Raistrickin **(66)**	*Penicillium*	−16.90	13.96	−22.09
Brevianamide F **(67)**	*Penicillium*	−9.31	−10.74	−12.92
*α*-Cyclopiazonic acid **(68)**	*Penicillium*	18.89	23.11	16.10
Terretrione A **(69)**	*Penicillium*	−18.30	−20.70	−24.36
Didymellamide A **(70)**	*Stagonosporopsis*	7.00	20.45	4.37
Thielaviazoline **(71)**	*Thielavia*	−9.52	−5.20	−12.09
Gymnastatin Z **(72)**	*Westerdykella*	**−34.15**	**−24.29**	**−34.28**

SARS-CoV-2 MPro ligand (FHR/PRD_002347)		−4.60	ND	ND
Main SARS-CoV-2 PL^pro^ ligand (Y97)		ND	−4.08	ND
Main SARS-CoV-2 3CL^pr^ ligand (3WL)		ND	ND	−34.66
Remdesivir		−35.56	2.28	−33.56

FD: fail to dock; ND: not done; positive values indicate unfavorable interactions.

**Table 2:** The absorption, distribution, metabolism, excretion, and toxicity (ADMET/TOPKAT) predictions for bioactive compounds, eutypellazine M **(57)**, scalusamide C **(62),** and gymnastatin Z **(72)** and the cocrystalized ligands with the examined proteins.

Compounds	Eutypellazine M	Scalusamide C	Gymnastatin Z	SARS-CoV-2 M^Pro^ ligand	SARS-CoV-PL^pro^ ligand	SARS-CoV-2 3CL^pr^ ligand
ADMET						
Absorption level	0	0	2	0	0	0
Solubility level	3	3	2	3	2	3
BBB level	3	2	4	4	0	3
PPB level	True	True	False	False	True	True
CPY2D6	NI	NI	NI	NI	Inhibition	NI
Hepatotoxic	Nontoxic	Nontoxic	Nontoxic	Nontoxic	Toxic	Toxic
PSA-2D	94.02	58.77	71.74	120.98	33.46	88.68
Alog p98	2.15	2.85	6.44	2.56	4.66	2.41

TOPKAT						
Ames prediction	Nonmutagen	Nonmutagen	Nonmutagen	Nonmutagen	Mutagen	Nonmutagen
Rat oral LD_50_ (g/kg.bw)	0.28	1.35	1.16	0.97	0.52	0.27
Rat female FDA	Noncarcinogen	Noncarcinogen	Noncarcinogen	Noncarcinogen	Noncarcinogen	Noncarcinogen
Rat male FDA	Noncarcinogen	Noncarcinogen	Noncarcinogen	Noncarcinogen	Noncarcinogen	Carcinogen
Skin irritancy	None	Moderate	Mild	Mild	None	None
Ocular irritancy	Severe	Moderate	None	Moderate	Mild	Mild
Rat chronic LOAEL(g/kg.bw)	0.03	0.08	0.18	0.21	0.02	0.15

0, 1, 2, and 3 indicate good, moderate, low, and very low absorption, respectively; 0, 1, 2, 3, 4, and 5 indicate extremely low, very low but possible, low, good, optimal, and too soluble, respectively; 0, 1, 2, 3, and 4 denote very high, high, medium, low, and undefined, penetration via BBB, respectively. PBB is plasma protein binding; FALSE means less than 90%; TRUE means more than 90%; NI is noninhibitor.

## Data Availability

Data are available in the manuscript.
